# Psoriasin (S100A7) is a novel biomarker for lung squamous cell carcinoma in humans

This article has been retracted.

**DOI:** 10.1186/s12935-014-0154-0

**Published:** 2015-02-12

**Authors:** Guijuan Liu, Qiang Wu, Guilan Liu, Xueying Song, Jihong Zhang

**Affiliations:** Department of Cytology Laboratory, People’s Hospital of Linyi, Linyi, 276300 Shandong China; Department of Nursing, People’s Hospital of Yinan, Linyi, Shandong 276300 China; Department of Nursing, People’s Hospital of Yinan, Linyi, Shandong 276300 China; Department of Thoracic Surgery, the People’s Hospital of Rizhao, Rizhao, China

**Keywords:** Lung squamous cell carcinoma, S100A7, NF-κB

## Abstract

**Objective:**

Psoriasin (S100A7) plays a role in the malignant potential of several epithelial cancers, and could candidate diagnostic marker or therapeutic target. Nuclear factor kappa B (NF-κB) regulates cancer cell growth and is modulated by phospholipase activity in many cancer cells. In the present study, we first evaluate the involvement of S100A7 in lung squamous cell carcinoma and its clinical usefulness for diagnosis. We then study whether knockdown of S100A7 in lung squamous cell carcinoma cells would reduce cell proliferation and NF-κB activity in vitro and attenuate tumor growth in vivo.

**Methods:**

We examined S100A7 expression in lung squamous cell carcinoma tissues by immunohistology. The human lung squamous cell carcinoma cell line NCI-H520 were transduced with short hairpin RNA targeting S100A7. Quantitative reverse transcriptase-polymerase chain reaction and immunoblotting confirmed knockdown of S100A7 messenger RNA and protein, respectively. Cell proliferation was evaluated by the MTT assay. NF-κB phosphorylation was assayed by western blot. 1 × 10^6^ of NCI-H520/S100A7 knockdown cells were injected into the left flanks of nude mice (aged 6 to 8 weeks). Tumors were followed for 35 days, then removed and stained with hematoxylin and eosin, stained with Ki-67, and analyzed for S100A7 protein expression.

**Results:**

S100A7 protein levels were significantly higher in carcinoma specimens than in nonneoplastic tissues. S100A7 might be a useful marker for diagnosis of lung squamous cell carcinoma. In vitro data showed that inhibition of S100A7 decreased proliferation of NCI-H520 cells. S100A7 knockdown reduced NF-κB phosphorylation and tumor growth in vivo and vivo. Explanted knockdown tumors maintained lower S100A7 levels compared with wild-type, confirmed by immunohistology. Ki-67 staining was more prominent throughout the wild-type tumors compared with knockdown tumors.

**Conclusions:**

Our present results suggest that S100A7 level is a promising tool for diagnosis of lung squamous cell carcinoma. Knockdown of S100A7 suppresses lung cancer growth in part by attenuating NF-κB activity. S100A7 may be a promising therapeutic target for lung squamous cell carcinoma.

## Introduction

Psoriasin (S100A7) is a small calcium binding protein of 11 kDa molecular weight. It is a member of the S100 family of the EF-hand type of calcium binding proteins. The S100A7 protein is known to be expressed in various tumors having squamous differentiation as a major component with or without accompanying inflammation [1-5]. Expression of both S100A7 mRNA and protein was also found in squamous cell carcinomas (SCC), adenosquamous carcinomas and large cell lung carcinomas, whereas neither was detected in adenocarcinomas or paired non-cancerous lung tissues. Further immunohistochemical analysis identified positive staining of S100A7 only in squamous cell carcinomas and large cell lung carcinomas, but not in other subtypes of lung cancer and normal lung tissues [6]. Recently, it has found S100A7 expression is closely associated with SCC metastasis to brain [7]. Taken together, the data suggest that S100A7 is promising diagnostic markers and/or therapeutic targets for SCC.

Although S100A7 has been reported to play a role in SCC, the molecular mechanisms of its effects are not well known. Nuclear factor kappa-B (NF-κB) transcription factors facilitate cell growth by stimulating proliferation genes. In cancer cells, breakdown of NF-κB feedback loops or constitutive activation of NF-κB leads to increased proliferation, angiogenesis, and metastasis [8]. NF-κB target genes include components of the arachidonic acid pathway [9] as well as proteins that increase the transcription of growth factors [10]. Evidence suggests that S100A7 modulates NF-κB levels in different cells [11,12], and both NF-κB and its target genes are downregulated when S100A7 is inhibited [11].

In the present study, we measured the expression of S100A7 in squamous cell carcinoma tissues by immunohistology and evaluated its clinical usefulness for diagnosis in SCC patient. We hypothesize that the knockdown of S100A7 in SCC cells will reduce cell proliferation and that this effect will correlate with decreased NF-κB activity. Furthermore, we propose S100A7 knockdown in SCC cells will attenuate tumor growth in vivo.

## Materials and methods

### Cell lines and reagents

NCI-H520 cells were from American Type Culture Collection. LC-2/ad cells were from RIKEN BRC. Cells were maintained in a humidified atmosphere with 5% carbon dioxide using Ham’s F-12 media (Cellgro, Manassas, Va) or Roswell Park Memorial Institute Media 1640 (Gibco, Grand Island, NY), respectively, with 10% fetal bovine serum (FBS). Tumor necrosis factor-alpha (TNF-α) was used to induce NF-κB activation. It was dissolved in phosphate buffered saline (PBS) and used at a concentration of 20 ng/mL. Antibodies for phosphorylated and total NF-κB and GAPDH were obtained from Cell Signaling Technology, Inc (Beverly, Mass). Antibody for S100A7 was obtained from Abcam (Cambridge, Mass).

### Patients and tissue collection

Surgically resected lung squamous cell carcinomas (SCC) tissues (n = 240) and specimens of normal lung adjacent to the tumor tissues (n = 60) were obtained from People’s hospital of Linyi, Shandong. Follow-up information was available for 143 cases. None of the patients had been treated with any preoperative chemotherapy or radiotherapy before surgery. After surgical resection, all patients received standard therapies according to the 2004 NCCN Clinical Practice Guidelines in Oncology for NSCLC. After cancer recurrence, the treatment was determined by individual physicians caring for their patients. Written informed consent was obtained from each patient, and institutional review board approval of this study was obtained from People’s Hospital of Linyi. The histological classification of these tumors was based on the WHO criteria [13]. Pathologic staging was done according to the tumor-node metastasis system for lung cancer staging [14].

### Immunohistochemical staining

Four-micron-thick TMA sections were used in all analyses. The sections were deparaffinized with xylene and rehydrated through graded alcohol incubations into water. They were then processed following the optimal staining protocol, as described above. In short, heat-induced epitope retrieval was performed using a Decloakig Chamber (DAKO, Kyoto, Japan), in which tissues were heated to 125°C then cooled to 90°C in Tris/EDTA buffer at pH 9 (Target Retrieval Solution; DAKO). After heat-induced epitope retrieval treatment, endogenous peroxidases were blocked with Peroxidase-Blocking Solution (DAKO) for 5 min. The sections were then incubated with anti-S100A4 antibody (1:50 dilution) for 60 min, followed by incubation with EnVision + Dual Link system, according to the manufacturer’s recommendations (DAKO). The reaction products were visualized with DAB+ (DAKO). All procedures were carried out at room temperature.

### Scoring of the Immunohistochemical staining

Semiquantitative evaluation of the sections was performed by 2 pathologists in a blinded manner. The negative control for immunostaining was performed without primary antibody. Both the fraction and intensity of the immunostained tumor cells were considered. The fraction score was calculated as the average of 5 randomly selected high-power fields assessed by light microscopy as follows: 0, no stained target cells (tumor, bronchial or alveolar cells); 1,20% of cells stained; 2, 20,50% of cells stained; and 3, over 50% of cells stained. The intensity score was defined as follows: 0, no appreciable staining of the target cells; 1, barely detectable staining in the cytoplasm and/or nucleus of the target cells; 2, readily apparent brown staining; and 3, dark brown staining. The fraction and intensity scores were multiplied to give a total score ranging from 0 to 9. Scores between 2 and 9 were regarded as positive expression. Immunohistochemical assays were also performed on histological sections of paraffin-embedded xenograft tumors.

Staining of the proliferative marker Ki-67 was performed to assess the growth of the xenograft tumors. The Ki-67 antibody (diluted 1:100) was obtained from Thermo Fisher Scientific, Rockford, USA. The Ki-67 labeling index (Ki-67 LI) was calculated according to the following formula: Ki-67 LI = number of Ki-67 positive cells/total number of tumor cells counted × 100%.

### Short-Hairpin RNA (shRNA) vectors

pUSE vectors containing non-targeted shRNA and 4 distinct shRNA sequences targeting S100A7 were purchased from Sigma-Aldrich. Cells were transfected with the appropriate expression construct, or control empty vector (pUSE), using Lipofect-AMINE 2000 (Invitrogen, Carlsbad, CA) in accordance with the manufacturer’s protocol. Stable clones were selected by continuous treatment with G418 (Life Technologies, 0.8 mg/mL) over 4 weeks.

### RNA extraction, cDNA synthesis and quantitative real time PCR

Total RNA was prepared from cultured cells using an RNeasy® Mini Kit (Qiagen, Maryland, USA), according to the manufacturer's protocol. cDNA was synthesized using SuperScript™II RNase H-Reverse Transcriptase (Invitrogen™, Sweden), as described by the manufacturer. The relative expression of S100A7 was analyzed using real-time PCR and the LightCycler instrument (Roche Applied Science, Sweden), together with the Light Cycler Fast Start DNA Master SYBR Green I kit (Roche Applied Science, Sweden), according to the manufacturer’s instructions. Primers for S100A7 [5] and β-actin [15] were as previously described. Two μl of cDNA were added to 18 μl of PCR Master Mixture (including 3 mM of MgCl2, 0.5 Mm of primers (S100A7 and β-actin) and 2 μl of LightCycler ™Fast Start Master SYBR Green). The protocol consisted of a 10-min denaturation step at 95°C and 40–45 cycles of amplification at 95°C for 10 seconds, 58°C (S100A7) and 60°C (β-actin) for five seconds and 72°C for eight seconds (β-actin) and 10 seconds (S100A7) respectively. After amplification, melting curves were obtained to verify the specificity of the amplification reaction and the products were also run on a 2% agarose gel. Quantitative analysis was performed with the LightCycler software version 3.5 (Roche Applied Science, Sweden), which estimates the crossing point (CP) for each sample. The CP values determined for psoriasin were normalized to β-actin (endogenous control).

### Western blotting

Cells were plated on 6-well plates at a density of 3 × 10^6^ in full media for 24 hours, then serum-starved (0.5% FBS) for 24 hours, then treated. Cells were stimulated with or without TNF-α (20 ng/mL) for 4 hours, then lysed with Laemelli buffer under reducing conditions. Time trials with TNF-α identified sustained changes in NF-κB activation at this time point (data not shown). Proteins were separated using sodium dodecyl sulfate polyacrylamide gel electrophoresis techniques and transferred to nitrocellulose membranes. Membranes were blocked in 5% nonfat milk in 1 × PBS, 0.1% Tween-20 (Sigma-Aldrich). Primary antibodies were dissolved in 5% bovine serum albumin (Sigma-Aldrich), 1 × PBS, 0.1% Tween-20. Secondary antibodies were prepared in 5% nonfat milk in 1 × PBS, 0.1% Tween-20. The protein of interest was developed using Pierce ECL Chemiluminescent (Thermo Fisher Scientific, Inc, Rockford, Ill). Densitometric analysis was performed using ImageJ Software (National Institutes of Health, Bethesda, Md).

### Cell proliferation assay

The cells were seeded onto 96-well plates at 4,000 per well in culture medium (100 μL). After culturing for 72 hr, cell numbers were measured by 3-(4,5-dimethylthiazol-2-yl)-2,5-diphenyltetrazolium bromide assay as described previously [16]. Briefly, 3-(4,5-dimethylthiazol-2-yl)-2,5-diphenyltetrazolium bromide (10 μL; 5 mg/mL) was added to each well and incubated for 4 hours at 37°C at 72 hr. The reaction was stopped by adding 100 μL of 0.04 N HCl in isopropanol to each well, with vigorous mixing to solubilize colored crystals produced by the reaction. The absorbance at 570 nm to absorbance at 630 nm as reference wave was measured by a multi well scanning spectrophotometer. Each data point is the average of six determinations and each experiment was repeated thrice.

### Xenograft experiment

All xenograft experiments were performed under a protocol approved by the People’s Hospital of Linyi, Animal Care and Use Committee. Male nude mice aged 6 weeks were purchased from Shandong University and quarantined for 2 weeks. At age 8 weeks the mice were injected into their left flanks with 1 × 10^6^ cells in 100 μL PBS. Flank tumors were measured every 2 to 3 days using digital calipers and volume was calculated by multiplying height × length × width. Xenograft tumors were removed en bloc and a portion from each tumor was preserved in 4% formalin in PBS and RNA later. Immunohistochemical staining of tumor tissue homogenate was used to examine S100A7 as described above. Tumors preserved in formalin were paraffin embedded; cut onto slides; and stained with hematoxylin and eosin, and for Ki-67. Histology was reviewed by a pathologist blinded to the study.

### Statistical analysis

SPSS 11.0 for Windows (SPSS Inc., Chicago, Ill, USA) was used for all data analysis. The immunohistochemical results and their associations with clinical characteristics were analyzed using the chi-square test. Spearman’s rank test was used to analyze the correlation between protein phenotypes. The Kaplan-Meier method was used to analyze univariate survival, and comparisons of the survival distributions among groups were performed using the log-rank test. The prognostic significance of S100A7 expression with respect to other pathological variables was assessed using multivariate Cox regression analysis. The quantitative data are expressed as the mean ± S.D. Student *t* test was performed for 2 group comparisons, and analysis of variance test was performed when comparing 3 or more groups. All *P* values were 2-tailed, and values of P < 0.05 were considered statistically significant.

## Results

### S100A7 is upregulated in SCC tumor tissues

S100A7 was prominently expressed in SCC (n = 140) in the cytoplasm of tumor cells (Figure 1). S100A7 level was significantly increased in SCC tissues compared with the normal lung tissues (*P* < 0.001) (Table 1).

**Figure 1:** **S100A7 is overexpressed in SCC tumor tissues.** Typical IHC staining images of human SCC tumor and normal lung tissue (magnification × 200).

**Table 1:** **Expression of S100A7 in SCC and normal lung tissue**

**Protein**	**Positive/Negative**	**SCC n= 143(100%)**	**Normal lung tissue n = 60 (100%)**	***P***
S100A7	Positive	87 (60.8%)	11 (18.3%)	<0.001
	Negative	56 (39.2%)	49 (81.7%)	

### Positive expression of S100A7 is associated with poor prognosis for SCC

Patients with complete clinical information were enrolled in the survival analysis. The median age was 61.00 years (range, 28.4 to 83.8 years). The clinical characteristics and survival analysis results are summarized in Table 2 and Figure 2. The 5-year survival rate for the entire group was 49.18 %, and the median follow-up time was 58.2.00 months (range, 0 to 78.02 months). Univariate analysis was performed to estimate the relation between clinical characteristics and S100A7 expression. As shown in Table 2, SCC patients with different clinical characteristics, such as sex, age, histological type and tumor-node-metastasis (TNM) stage, demonstrated similar levels of S100A7. No relationship was found between S100A7 expression and metastasis.

**Table 2:** **Clinical characteristics of patients, S100A7 expression and the survival analysis**

	**S100A7 experssion**			**Log rank**	**Median**	**Log rank**	**Cox regression**					
**Factors**	**+(n)**	**-(n)**	***P***	**Total**	**Survival**	**Subgroup**	**Univariate**			**Multivariate**		
				***P***	**(Months)**	***P***	**HR**	**95 % CI**	***P***	**HR**	**95% CI**	***P***
**Gender**			0.304	0.274								
Female (n = 38)	14	24			57.12	0.075						
Male (n = 105)	63	42			59.20	0.024						
**Age**			0.29	0.451								
<60y (n = 49)	30	19			59.13	0.146						
≧60y (n = 94)	57	37			52.24	0.018						
**Tumor size**			0.014	0.000								
T1+T2 (n = 92)	71	21			62.3	0.0026	2.128	1.38-3.472	0.002	1.563	1.028-2.859	0.047
T3+T4 (n = 51)	16	35			36.2	0.437						
**Differentiation**			0.473	0.269								
Low (n = 94)	62	32			52.8	0.016						
Moderate/high (n = 49)	25	24			60.5	0.162						
**Lymph node**			0.063	0.000			2.846	1.93-5.053	0.001	2.73	1.40-3.180	0.02
N0+N1 (n = 106)	69	37			61.5	0.012						
N2+N3 (n = 37)	18	19			30.8	0.165						
**Distant M**			0.258	0.684			1.235	0.63-2.158	0.392			
M0 (n = 131)	79	52			59.6	0.006						
M1(n = 12)	8	4			44.8	0.538						
**Clinical stage**			0.082	0.0013			2.35	1.364-3.86	0.001	0.93	0.435-1.132	0.876
I+II(n = 89)	49	40			615	0.038						
III+IV(n = 54)	38	16			37.9	0.026						
**S100A7 (n = 143)**	87	56	0.001	0.007	58.2/43.8		1.926	1.23-3.28	0004.	2.01	1.35-4.157	0.002

**Figure 2:** **Positive expression of S100A7 is associated with poor prognosis for SCC.** Patients with positive S100A7 expression had shorter survival times, *P* = 0.008.

The prognostic significance of positive S100A7 expression in different subgroups was assessed using the log rank test. In the entire group, patients with positive S100A7 expression had shorter survival times (Figure 2, *P* = 0.008). The results also indicated that male sex, older age and positive S100A7 expression were associated with worse prognosis (Table 2). Moreover, multivariate Cox regression analysis revealed that tumor size, lymph node invasion and S100A7 expression were independent predictors of SCC prognosis (Table 2). These results suggested that S100A7 plays an important role in SCC tumorigenesis and prompted further analysis.

### Knockdown of S100A7 in NCI-H520 cells

NCI-H520 cells were stably transduced with green fluorescent protein-tagged pUSE vector particles to confirm efficacy of technique and optimal concentration of particles for transduction (Figure 3A). Cells were then transduced with pUSE shRNA S100A7 for S100A7, or nontargeted shRNA as a control. Selection for transduced cells was with puromycin antibiotic. A kill curve was performed to determine a puromycin concentration of 2 μg/mL for selection (data not shown). Four distinct short hairpin sequences targeting S100A7 were used and examined for knockdown of S100A7 both mRNA and protein expression. RT-PCR confirmed decreased mRNA with all sequences, from S1 to S4 (Figure 2B). Western blot for S100A7 revealed sequence S4 resulted in the most robust knockdown of protein expression (Figure 3C). All subsequent experiments used NCI-H520 cells transduced with sequence S4 shRNA targeting S100A7, or nontargeted shRNA, compared. with nontransduced wild-type NCI-H520 cells.

**Figure 3:** **Knockdown of S100A7 in NCI-H520 cells.** Short-hairpin RNA (shRNA) sequence S4 obtains most robust knockdown of S100A7 messenger RNA and protein. ANCI-H520 cells were stably transduced with green fluorescent protein (GFP)-tagged pUSE shRNA, **(A)** to determine the optimal conditions for transduction, before transducing cells with vector particles containing nontargeted shRNA as a control, or shRNA targetingS100A7. Growth selection for transduced cells was with puromycin. Four distinct shRNA sequences (S1 to S4) targeting groupS100A7 were used to create 4 different knockdown cell lines. **(B)**. Knockdown was confirmed by messenger RNA and **(C)** protein analysis. The most robust knockdown in protein was with sequence S4.

### S100A7 knockdown inhibits proliferation in ANCI-H520 cells

Stable knockdown of S100A7 mRNA compared with both wild-type controls and nontargeted controls was confirmed over several cell passages using RT-PCR (Figure 4A). Proliferation studies using the 5-bromo-2′-deoxyuridine assay were performed with the same passages of cells. Results showed a stable reduction by approximately 48% in the growth rate of NCI-H520 knockdown cells compared with both control groups (Figure 4B). This is consistent with our finding during cell culture that double the concentration of S4 cells compared with nontargeted or wild-type cells were required for the cells to reach confluence at the same time (data not shown).

**Figure 4:** **S100A7 knockdown inhibits proliferation in ANCI-H520 cells.** S100A7 knockdown is stable over several cell passages with corresponding persistent decrease in growth rate of lung cancer cells. **A**. Quantitative reverse-transcription polymerase chain reaction confirms decreased messenger RNA (mRNA) over several cell passages 1 through 7. **B**. Analysis of proliferation using the same cell passages 1 through 7 shows a stable reduction in the growth rate of NCI-H520 knockdown cells. Controls for the experiments are wild-type cells and vector controls (NT). Data are presented as mean ± standard error of the mean; n =3 performed in triplicate. *P < 0.05.

### S100A7 knockdown decreases NF-κB activity

Results show TNF-a treatment induces NF-κB phosphorylation. However, NF-κB phosphorylation in S4 cells is significantly decreased compared with nontargeted or wild-type cells (Figure 5).

**Figure 5:** **S100A7 knockdown decreases NF-κB activity.** S100A7 knockdown decreases nuclear factor-κB (NF-κB) activity. Tumor necrosis factor-α (TNF-α) induces NF-κB phosphorylation in NCI-H520 cells, vector control cells (NT) and knockdown cells (S4), though significantly less in the knockdown cells. Representative Western blot of a single experiment is shown with a graph of densitometric analysis of cumulative experiments below (mean ± standard error of the mean; n = 5 per group). *P < 0.05.

### S100A7 knockdown decreases NCI-H520 xenografts growth in vivo

Xenografts of S4 cells grew significantly slower than wild-type cells or vector control cells (*NT*) (Figure 6A), with wild-type tumors growing to double the volume of knockdown tumors at post injection day 35. Tumors were also stained with Ki-67, a marker of proliferation. Wild type tumors had more Ki-67 staining and the location of the staining was throughout the tumor, compared with knockdown tumors where the staining was more visible at the periphery (Figure 6B). Analysis of S100A7 expression in xenograft tumors confirmed persistent decrease in S100A7 in knockdown tumors compared with wild-type tumors (data not shown).

**Figure 6:** **S100A7 knockdown decreases NCI-H520 xenografts growth in vivo.** NCI-H520 and knockdown cells were injected into the left flanks for nude mice and tumor size was serially measured until post injection day 35. **A**. Volume of the tumors over time shows significant growth retardation in the knockdown cells (S4) compared with NCI-H520 or vector control cells (*NT*) cells (mean ± standard error of the mean; n = 6) per group. **B**. wild-type tumors exhibit increased Ki-67 expression compared with the knockdown tumors. (^*^ *P* < 0.05).

## Discussion

The S100 gene family encodes small proteins that share EF-hand helix-loop-helix domains that are important for their function as calcium-binding proteins [17]. Several S100 genes are altered in neoplasia including S100A7. S100A7 was first identified as a highly abundant cytoplasmic and secreted protein that is induced in abnormally differentiating squamous epithelial cells derived from epidermis of skin affected by psoriasis [18]. This association with psoriasis has suggested a role for S100A7 either in keratinocyte differentiation or as a chemotactic factor [19-21].

It has since been found to be expressed in association with neoplasia in several tissues including squamous carcinomas of the head and neck, the cervix and the lung [18], the skin [22], the bladder [23], as well as adenocarcinomas of the stomach [24] and the breast [5,25]. From the study of S100A7 expression at different stages of progression in both the skin and the breast, it is clear that while the protein is not generally expressed in normal epithelia, an increasing frequency of expression is seen beginning with early stages of progression [22,26].

Recently, a number of studies have shown that SCC can positively regulate the proliferation and apoptosis of tumor cells, although the precise role of S100A7 in lung cancer remains unknown. Therefore, the current study explored the prognostic significance of S100A7 and its function in SCC. In our study, we found overexpression of S100A7 in SCC tissues was observed when comparing SCC tissues with adjacent normal tissues, and this aberrant accumulation of S100A7 in SCC cells was associated with a shorter survival time and identified as a novel risk factor for poor prognosis. Although little attention has been paid to the expression of S100A7 in lung cancer, evidence suggests that the overexpression of S100A7 may serve as a marker for worse prognosis in SCC.

This is the first study that demonstrates decreased proliferation and tumor growth in vivo and vitro with knockdown of S100A7 mRNA. RNA interference is a potential therapeutic tool. Given that short hairpin knockdown of S100A7 mRNA slows tumor growth, targeted RNA interference of S100A7 may have a therapeutic application in the treatment of SCC.

Although analysis of S100A7 expression has been reported, the role of S100A7 is not well understood. In the present study, RNAi experiments clearly showed that S100A7 is involved in cell proliferation of lung cancer cells. Our RNAi data revealed that inhibition of S100A7 affects expression of NF-kB activation, which are involved in cell proliferation. The results demonstrated a dominant link between NF-κB, S100A7, and cell viability. Our study shows that knockdown of S100A7 decreases NF-κB activity, further supporting the hypothesis of a role for S100A7 and NF-κB interaction that slows tumor growth. These data suggest not only potential for S100A7 as a therapeutic target, but also several mechanisms that can be examined to better understand the unique role of S100A7 in lung tumor growth. Targeting S100A7 may exploit its relationship with NF-κB because NF-κB target genes include transcription factors for a number of growth factors such as vascular endothelial growth factor, fibroblast growth factor, and platelet-derived growth factor, which have been linked to promoting cancer cell growth, tumor stroma development, and angiogenesis [27-29].

Another hallmark of cancer is its activating mechanisms of invasion and metastasis [30]. In our 143 patients, no relationship was found between S100A7 expression and metastasis. Further studies will better address the role of S100A7 in metastatic disease in vivo and vitro.

In conclusion, S100A7 has significant value to predict postoperative recurrence and overall survival of patients with SCC. Disclosing the genes regulated by S100A7 will provide further clues to its biological roles and more generally will contribute to the understanding of the mechanisms underlying the growth of lung cancer. Interestingly, S100A7 plays a significant role in modulating lung cancer cell growth. The relevance of S100A7 as a therapeutic target has expanding potential and studies investigating the expression of S100A7 in human tumor tissue are ongoing.
